The article "Analysis of the Relationship between Gut Flora Levels in Childhood Obese Population and Normal Healthy Population Based on Machine Learning" was retracted in 2023. Reasons: signs of a paper mill; compromised peer review; unreliable results or conclusions.

# Analysis of the Relationship between Gut Flora Levels in Childhood Obese Population and Normal Healthy Population Based on Machine Learning

**DOI:** 10.1155/2022/6860940

**Published:** 2022-08-28

**Authors:** Yaoqing Feng, Xia Si, Ruifang Zhu, Junxiang Chen, Wenting Zhao, Qian Wang, Shifan Han

**Affiliations:** School of Nursing, Shanxi Medical University, 56 Xinjian South Road, Taiyuan, Shanxi Province 030001, China

## Abstract

**Aims:**

To explore the study of the relationship between the level of gut flora in childhood obese people and normal healthy people based on the analysis of machine learning.

**Materials and Methods:**

The stools of 54 normal weight, 53 overweight, and 59 obese children from May 2021 to May 2022 were selected. And DNA was extracted, and primers specific for the four bacteria were designed according to the specificity of the four bacteria to the 16 S rDNA gene sequences of the bacteria to be tested, and real-time fluorescence quantitative PCR reactions were performed to compare whether there was any difference in the number of the four bacteria between the three groups*. Results*. The results of agarose gel electrophoresis showed that the PCR amplification products of all four target bacteria showed clear bands at the corresponding positions, and no nonspecific bands appeared. When compared with the marker, the size matched with the target fragment, indicating good primer specificity. The comparison between normal body recombinant, super recombinant, and obese groups was statistically significant (*P* < 0.05) for rectal eubacteria, polymorphic anaplasma, bifidobacteria spp., and lactobacilli. The median number of bifidobacteria in the three groups was significantly higher than the median number of rectal eubacteria, polymorphomycetes, and lactobacilli. The difference in comparison was statistically significant (*P* < 0.05). Stratified analysis of children's age revealed that normal body composition of Lactobacillus decreased with increasing age, and the difference was statistically significant (*P* < 0.05).

**Conclusion:**

An increase in rectal eubacteria and a decrease in polymorphomycetes, bifidobacteria spp., and lactobacilli may be associated with the development of obesity. The numbers of rectal eubacteria, polymorphic methanobacteria, bifidobacteria spp., and lactobacilli in the intestine of normal weight and obese children were less affected by sex and age.

## 1. Introduction

With the development of the economy and the improvement of people's living standards, in the past three decades, the three indicators of body mass index, prevalence of obesity, and prevalence of overweight individuals have increased significantly worldwide. Health risks have received extensive attention from researchers around the world [1]. Prevention and treatment of obesity and related complications have been shown to be lengthy and complex, and successful strategies for treating obesity remain limited. Epidemiological studies have revealed potential environmental factors that affect obesity, including diet, energy expenditure, lack of sleep, endocrine disorders, chronic inflammation, and microbiome status, which may lead to an increased risk of obesity [2].

The article "Analysis of the Relationship between Gut Flora Levels in Childhood Obese Population and Normal Healthy Population Based on Machine Learning" was retracted in 2023. Reasons: signs of a paper mill; compromised peer review; unreliable results or conclusions.

Under normal circumstances, the intestinal flora maintains a dynamic balance with the internal and external environment of the human body. Once this balance is broken, intestinal microbial structural imbalance will occur, which will lead to the occurrence and development of obesity and related metabolic diseases. Studies have shown that Firmicutes are closely related to obesity because they can better assist the body to absorb energy from the external environment [3]. In recent years, the relationship between intestinal flora and diseases has attracted extensive attention from scholars at home and abroad, and many new research ideas have been proposed, some of which have also made breakthroughs [4]. However, there are still few studies on the relationship between gut microbiota and children of different weights, especially the relationship between overweight and obese children and some specific microbiota [5]. In order to reasonably integrate and correlate massive data with relevant biological information, so as to better serve practical applications, researchers have introduced machine learning methods into the analysis of gut microbiota data as early as six years ago [6]. Compared with classical statistical methods, machine learning is more suitable for dealing with large-scale learning problems and shows excellent performance when dealing with high-dimensional structured data obtained by metagenomic sequencing [7]. Machine learning methods can deeply mine the interaction information contained in the flora data by extracting features, which can deal with a variety of biological information problems, identify relevant biomarker variables based on sparse data, and prevent overfitting [8]. For multitask problems, the performance is improved by using information from various related tasks, for clustering feature analysis of unlabeled data [9]. We studied the characteristics of intestinal flora changes in obese children and explored the relationship between intestinal flora and obesity, in order to provide a theoretical basis for the prevention and treatment of obesity by regulating intestinal flora.

## 2. Material and Methods

### 2.1. Research Object

Stools of 54 normal weight, 53 overweight, and 59 obese children were selected from May 2021 to May 2022. Normal weight children and overweight and obese children were screened strictly according to the predefined inclusion and exclusion criteria, and fresh stools were collected using disposable stool collection tubes and stored at -80°C.

The article "Analysis of the Relationship between Gut Flora Levels in Childhood Obese Population and Normal Healthy Population Based on Machine Learning" was retracted in 2023. Reasons: signs of a paper mill; compromised peer review; unreliable results or conclusions.

### 2.2. Inclusion and Exclusion Criteria

Inclusion criteria are as follows: (i) aged between 6 and 11 years old; (ii) meeting the criteria for determining normal weight, overweight, and obesity in children; comparison of BMI (kg/m^2^) cut-off points [10] (see Table 1); and (iii) willing to participate in the study and obtain the consent of the guardian, voluntarily serve as the subject, and sign the informed consent. Exclusion criteria are as follows: (i) antibiotic use in the past 4 weeks; (ii) gastrointestinal disorders, past history of gastrointestinal disease or diarrhea, bloating, abdominal pain or constipation within the past 4 weeks, trauma, serious infection, and infectious disease; and (iii) hereditary obesity, drug-induced obesity, endocrine disorders, and metabolic diseases.

### 2.3. Methods

#### 2.3.1. Fecal Genomic DNA Extraction

Weigh 200 mg of feces into a 2 ml centrifuge tube and place the tube on ice. Add 1.4 ml GSL to the centrifuge tube and shake intermittently for 1 min until the sample is well mixed. Incubate at 70°C for 5 min. Vortex for 15 seconds and centrifuge at 12000 pm for 1 minute. Pipette 1.2 ml of supernatant into a new 2 ml centrifuge tube. Take an inhibitor adsorbent tablet and add it to the supernatant, and shake it sufficiently to completely disperse and suspend the adsorbent tablet. Place at room temperature for 1 minute to promote the full effect of the adsorption sheet. Centrifuge at 12000 rpm for 3 minutes. Transfer the supernatant to a new 1.5 ml centrifuge tube and centrifuge again for 3 min. Transfer 200 *μ*l of the supernatant to a new 1.5 ml centrifuge tube, then add 15 *μ*l proteinase K and 200 *μ*l GB, and vortex for 15 seconds. Incubate at 70°C for 10 minutes. After a brief centrifugation, add 200 absolute ethanol. Vortex to mix and briefly centrifuge again. The solution was transferred to an adsorption column and centrifuged at 12000 pm for 30 seconds, and the waste liquid was discarded. Add 500 *μ*l GD, centrifuge for 30 seconds, and discard the waste liquid. Add 600 lPW, centrifuge for 30 seconds, then discard the waste liquid, and repeat the operation step 14. Centrifuge at 12000 pm for 2 minutes and discard the waste liquid. Place at room temperature for about 10 minutes to allow the residual liquid in the adsorbent material to dry. Put the adsorption column into a new 1.5 ml centrifuge tube, then add 50 *μ*l TB dropwise to the middle of the adsorption membrane, place it at room temperature for 5 minutes, and then centrifuge for 2 minutes. The solution in the centrifuge tube is the extracted DNA.

The article "Analysis of the Relationship between Gut Flora Levels in Childhood Obese Population and Normal Healthy Population Based on Machine Learning" was retracted in 2023. Reasons: signs of a paper mill; compromised peer review; unreliable results or conclusions.

#### 2.3.2. Agarose Gel Electrophoresis of PCR Products

Add 20 ml of TBE (50×) to 980 ml of double-distilled water, and dilute to TBE (1×) for later use; weigh 1 g of agarose powder, add 100 l of TBE (1×), and shake gently. Heat in a microwave oven until the agarose is completely melted, cool to about 60°C, add 10 *μ*l of GelRed dye, mix well, and pour it into the plastic plate with the comb inserted. After the gel has solidified, take out the comb, put the gel block into the electrophoresis tank, and add TBE (1×) buffer until the gel plate is covered. The DNA sample and loading buffer (6×) were mixed at a ratio of 5 : 1 and added to the sample well, and finally, the same volume of DNA marker was added. Turn on the power for electrophoresis, 120 V, 30 min. After the electrophoresis is completed, take pictures with a gel imaging analyzer. Under UV light, the band containing the target DNA was excised into a clean 1.5 ml centrifuge tube and weighed. According to the weight of the gel, the sol solution PN was added to the centrifuge tube in proportion (100 *μ*l of PN solution was added to 0.1 g of the gel) and heated in a 50°C water bath until the gel block was completely dissolved. Put the adsorption column into the collection tube, transfer the solution to the adsorption column, leave it at room temperature for 2 minutes, centrifuge at 12000 pm for 60 seconds, drain the waste liquid in the collection tube, then put the adsorption column back into the collection tube, add 600 l of rinse solution Centrifuge at PW.12000 pm for 1 minute, discard the waste liquid, and put the adsorption column back into the collection tube. Centrifuge again for 3 minutes. After centrifugation, the adsorption column was left at room temperature for 10 minutes. Put the adsorption column into a new 1.5 l centrifuge tube, then add 50 *μ*l of elution buffer TB dropwise to the middle of the adsorption membrane, leave it at room temperature for about 5 minutes, and centrifuge for 2 minutes. The solution in the centrifuge tube is the recovered gel. UV spectrophotometer detects the concentration: the DNA recovered from the above-mentioned cutting gel is used as the standard, and the concentration is detected by the UV spectrophotometer and converted into the corresponding copy number according to the formula: copy number = concentration (nggL) × 109 × 6.02 × 1031 (660 × the number of bases of the target gene). Preparation of standard curve: serially dilute each standard 10 times to form 10-10 copies/*μ*l, and carry out real-time fluorescence quantitative PCR reaction. To avoid systematic and manual errors, three replicate wells were made for each concentration of standard template. Real-time fluorescent quantitative PCR reaction system 20 *μ*: DNA template 1 *μ*l, upstream and downstream primers each 1 *μ*l, 2×RealStar Green Fast Mixture (with Rox) 10 *μ*l, and ddH_2_O 7 *μ*l. The amplification conditions of real-time quantitative PCR reaction were as follows: 95°C predenaturation for 2 minutes; 95°C denaturation for 15 s, Tm annealing for 30 s, 72°C extension for 30 s, 40 cycles; melting curve: 60°C to 95°C for each 0.3°C temperature increase to collect fluorescence. After the reaction, the StepOne software automatically draws a standard curve.

The article "Analysis of the Relationship between Gut Flora Levels in Childhood Obese Population and Normal Healthy Population Based on Machine Learning" was retracted in 2023. Reasons: signs of a paper mill; compromised peer review; unreliable results or conclusions.

### 2.4. Statistical Analysis

The SPSS 27.0 statistical software was used for analysis. Count data were expressed as the number of cases, and differences between the three groups were compared using chi-square test. If the measurement data obeyed normal distribution and the variance between the groups was the same, the data were expressed as mean ± standard deviation, and the differences between groups were compared using one-way ANOVA, and if the sample data did not meet several conditions mentioned above, the data were expressed as median/interquartile spacing, and the comparison between the three groups was done using multiple independent sample our rank sum test (Alaska-Wallis *H* test) with the test level *a* = 0.05.

## 3. Results

### 3.1. Electrophoresis of PCR Products

The results of agarose gel electroplate showed that the PC amplification products of the four target bacteria all showed clear bands at the corresponding positions, and no nonspecific bands appeared. When compared with the marker, the size matched with the target fragment, indicating good primer specificity (see Figure 1).

### 3.2. Differences in the Amount of Bacteria between Groups

The comparison of antibacterial rectum, Bacteroides polymorpha, Bifidobacterium, and Lactobacillus among the normal weight, overweight, and obese groups was statistically significant (*P* < 0.05). The median of Bifidobacterium in the three groups was significantly higher than that of antibacterial rectum, Bacteroides polymorpha, and Lactobacillus. The difference was statistically significant (*P* < 0.05) (see Figure 2).

### 3.3. Distribution Characteristics of Gut Microbiota in Different Genders

The gender stratified analysis of children showed that there was no significant difference in the distribution of intestinal flora among normal weight children, overweight children, and obese children (*P* > 0.05) (see Figure 3).

The article "Analysis of the Relationship between Gut Flora Levels in Childhood Obese Population and Normal Healthy Population Based on Machine Learning" was retracted in 2023. Reasons: signs of a paper mill; compromised peer review; unreliable results or conclusions.

### 3.4. Distribution Characteristics of Gut Microbiota at Different Ages

The stratified analysis of children's age showed that the normal body weight Lactobacillus decreased with the increase of age, and the difference was statistically significant (*P* < 0.05), and the other differences were not statistically significant (*P* > 0.05) (see Figure 4).

## 4. Discussion

The intestinal flora is closely related to human health. With the deepening of the research on the intestinal flora, people have realized that the intestinal flora plays an important role in the process of energy intake, transformation, and storage [11]. More and more studies have found that the intestinal flora has a certain relationship with the occurrence and development of obesity. Therefore, an in-depth study of the relationship between the changes in the intestinal flora and obesity, especially the relationship between specific bacteria and obesity, can be used for obesity prevention and development. Treatment offers new directions [12]. Studies on the relationship between gut microbiota and obesity have mainly focused on the phylum level. Studies in both animals and humans have found that compared with the control group, the obese individuals have an increase in Firmicutes and a decrease in Bacteroidetes or Firmicutes/Pseudobacterium The proportion of Bacillus phyla increased [13]. Based on this, our study is aimed at exploring the relationship between specific bacteria and obesity through quantitative research on specific bacteria [14]. Eubacterium rectum is a representative bacteria in the Firmicutes phylum, with the role of fermenting glucose or protein [15]. Eubacterium rectum contains genes related to resistant starch-degrading enzymes, which can reduce glycan-degrading enzymes, thereby increasing the expression process of selective amino acid and sugar transport, reducing the level of nicotinamide adenine dinucleotide (NADH), and promoting sugar fermentation [16]. Therefore, we have reason to think that Eubacterium rectum may be related to the host's energy metabolism. Bacteroides polymorpha is one of the most studied bacteria in the phylum Bacteroidetes. Because it contains 64 enzymes related to the degradation of polysaccharides, it has a strong ability to digest polysaccharides [17]. At the same time, it can hydrolyze and ferment exogenous fibrous substances and endogenous mucin to provide energy for the host [18]. Bacteroides polymorpha can also regulate and maintain the intestinal microecological balance by synthesizing vitamins, preventing the colonization of foreign bacteria, and enhancing the body's immunity [19]. Based on the characteristics of Eubacterium rectum and Bacteroides polymorpha, it can be speculated that changes in their numbers are closely related to obesity [20]. Probiotics refer to microorganisms that can benefit health after consumption, and the probiotics that exist in the human gut can also exert their beneficial effects by improving the intestinal microecological balance of the body. Bifidobacterium and Lactobacillus are the two most common probiotics [21]. On the one hand, the probiotic effect of bifidobacteria is to enhance the adsorption of intestinal mucosa by producing extracellular polysaccharides and colonize the surface of intestinal epithelial cells, thereby preventing the colonization of pathogens or opportunistic pathogens [22]. On the other hand, lactic acid and acetic acid are produced by decomposing carbohydrates, which makes the intestinal tract an acidic environment, thereby inhibiting the growth of spoilage bacteria and maintaining the microecological balance in the intestinal tract [23]. Lactobacillus is named because it can ferment sugars to produce lactic acid, so it can regulate intestinal microecology like Bifidobacterium [24]. Lactobacillus also has a role in regulating immune function, but there are relatively few studies on weight control [25].

The article "Analysis of the Relationship between Gut Flora Levels in Childhood Obese Population and Normal Healthy Population Based on Machine Learning" was retracted in 2023. Reasons: signs of a paper mill; compromised peer review; unreliable results or conclusions.

Our study found that the number of Eubacterium rectum in the overweight and obese children was significantly higher than that in the normal weight group, and the number of Eubacterium rectum in the obese group was significantly higher than that in the overweight group. It is speculated that it may lead to obesity by increasing energy absorption [26]. Some scholars have found that compared with normal mice, germ-free mice can absorb dietary glucose and metabolize starch but lack the complex fiber for digestion, so they cannot obtain energy from indigestible polysaccharides [27]. This indicates that certain gut microbiota can lead to obesity by increasing energy acquisition from polysaccharide diet [28]. Eubacterium rectum may be one of these bacteria [29]. Bacteroides polymorpha belongs to the phylum Bacteroidetes, is a Gram-negative bacterium, and is one of the most important bacteria in the human body [30]. Some scholars have found that ordinary people contain about 30% of Bacteroides in the intestine, while only 3% of Bacteroides in obese people increased to 15% [31]. The same is true for studies in mice, where obese mice had less Bacteroides than wild-type mice when fed the same low-fat diet but increased Bacteroides when they lost weight [32]. However, some scholars have found that the number of Bacteroides in the intestine of obese people is significantly higher than that of the lean group, but considering that the method of in vitro culture combined with microscopy is used and the number of people in the study is small, it is impossible to make a firm conclusion on the results [33]. Some scholars found that the real-time fluorescence quantitative PC technology was used to quantify B. polymorpha in patients with type 2 diabetes and normal control groups and found that the number of B. polymorpha in the type 2 diabetes group was lower than that in the normal control group [34]. In the study of hypertension, the hypertensive group was significantly lower than the normal control group, and some scholars found that the use of Bacteroides polymorpha gavage in mice found that it has a weight loss effect [35]. A further study in obese patients found that the number of B. polymorpha in the gut could be restored to normal weight levels by bariatric surgery [36]. Both animal and human studies have demonstrated that the reduction of B. polymorpha is associated with obesity.

The article "Analysis of the Relationship between Gut Flora Levels in Childhood Obese Population and Normal Healthy Population Based on Machine Learning" was retracted in 2023. Reasons: signs of a paper mill; compromised peer review; unreliable results or conclusions.

Our study found that the number of B. polymorpha in children with overweight and obesity was significantly higher than that in children with normal weight, but the difference between overweight and obesity groups was not statistically significant, indicating that the reduction of B. polymorpha may lead to the occurrence of overweight and obesity, but the specific mechanism is still unclear, and further research is needed. In our study, the four types of intestinal bacteria were stratified by gender and age among the three groups and found that the normal weight Lactobacillus decreased with the increase of age, and the difference was statistically significant. It indicated that the number of Lactobacillus in the normal body group was related to age, and the number of four bacteria in the other groups had nothing to do with age and gender. This is similar to the conclusion found in studies elsewhere in China that the distribution of gut microbiota in school-age children is less affected by children's gender and age. Lactobacillus is also a probiotic, which can ferment carbohydrates to produce a large amount of lactic acid, and is one of the important physiological flora of human [37]. In addition to improving immunity, anti-inflammatory, anticancer, etc., it also plays an important role in regulating intestinal flora [38]. A study found that the body weight and adipose tissue weight of mice fed with Lactobacillus were significantly lower than those in the control group, suggesting that Lactobacillus may control the growth of fat cells [39]. Studies have also found that Lactobacillus can significantly reduce abdominal fat and weight loss in obese mice, presumably by reducing fat absorption and affecting energy metabolism [40]. A number of epidemiological studies have found that cesarean section is a risk factor for childhood obesity. At the same time, some studies have pointed out that the intestinal tract of newborns born by cesarean section is mainly Lactobacillus, while the newborns born by cesarean section are mainly Staphylococcus and Acinetobacter [41]. Bifidobacterium belongs to Actinobacteria and is an important probiotic with the functions of improving immunity, antitumor, and antiaging and regulating intestinal flora [42]. It mainly regulates the intestinal flora through two aspects: on the one hand, by producing extrabacterial polysaccharides to enhance the adsorption to the intestinal mucosa and colonize the surface of intestinal epithelial cells, thereby preventing the colonization of pathogens or opportunistic pathogens [43]. On the other hand, by decomposing carbohydrates to produce lactic acid and acetic acid, the intestinal environment is acidic, thereby inhibiting the growth of spoilage bacteria [44]. Our study found that the number of Bifidobacterium in the obese group was significantly lower than that in the normal weight and overweight group, but the difference between the normal group and the overweight group was not statistically significant, indicating that the reduction of Bifidobacterium may be related to the occurrence of obesity [45]. The possible mechanism is that the reduction of bifidobacteria promotes the increase of harmful bacteria and destroys the stability of the intestinal mucosa, thereby unbalanced the absorption and metabolism of nutrients, leading to the occurrence of host obesity [46].

The article "Analysis of the Relationship between Gut Flora Levels in Childhood Obese Population and Normal Healthy Population Based on Machine Learning" was retracted in 2023. Reasons: signs of a paper mill; compromised peer review; unreliable results or conclusions.

We have a small amount of research samples, and there are certain limitations. All the data in our experiments are relatively concentrated and underrepresented. The detection of only four intestinal species that may be related to obesity cannot represent the entire intestinal microbes. It is hoped that more bacteria will be screened in the future to provide more support for obesity research. Our study is a preliminary exploration of the relationship between gut microbiota and overweight and obesity, and other technical means are needed to conduct mechanism research to comprehensively describe the relationship between gut microbiota and overweight and obesity. In conclusion, the increase of Eubacterium rectum and the decrease of Bacteroides polymorpha, Bifidobacterium, and Lactobacillus may be related to the occurrence and development of obesity. Quantities of Eubacterium rectum, Bacteroides polymorpha, Bifidobacterium, and Lactobacillus in the gut of normal weight and obese children were less affected by sex and age.

The article "Analysis of the Relationship between Gut Flora Levels in Childhood Obese Population and Normal Healthy Population Based on Machine Learning" was retracted in 2023. Reasons: signs of a paper mill; compromised peer review; unreliable results or conclusions.

## Figures and Tables

**Figure 1:** PCR product electroplate results (M: marker; 1, 2: rectal antibacterial; 3, 4: polymorphomycetes; 5, 6: Bifidobacterium spp.; 7, 8: Lactobacillus).

**Figure 2:** Differences in genus amounts between groups. In our study, data on differences in genus amounts between groups were statistically analyzed and calculated using the SPSS 27.0 statistical software. The measured data were expressed as median, and analysis of variance using repeated measures showed that rectal bacteria, polymorphic mimics, bactericidal spp., and bacilli were statistically significant (*P* < 0.05) when compared between the normal body recombination, super recombination, and obesity groups. The median number of bactericidal in the three groups was significantly higher than the median number of rectal bacteria, polymorphomycetes, and bacilli. The difference in comparison was statistically significant (*P* < 0.05).

**Figure 3:** Characteristics of intestinal flora distribution among different genders of children. In our study, data on the characteristics of intestinal flora distribution among different genders of children were statistically analyzed and calculated using the SPSS 26.00 statistical software. The measured data were expressed as median, and the analysis of variance using repeated measures showed that the differences were not statistically significant (*P* > 0.05) when comparing the intestinal flora distribution characteristics of normal weight children, overweight children, and obese children, stratified by gender.

**Figure 4:** Comparison of intestinal flora distribution characteristics at different ages. In this study, statistical analysis of data on intestinal flora distribution characteristics at different ages was calculated using the SPSS26.00 statistical software. The measured data were expressed as mean ± standard deviation, and repeated measures ANOVA showed that stratified analysis of children's age revealed that normal body composition of Lactobacillus decreased with increasing age and the difference was statistically significant (*P* < 0.05); the rest of the differences were not statistically significant (*P* > 0.05).

**Table 1:** Comparison of different BMI cut-off points for children and adolescents aged 6-11 years in China.

Age (years)				
	Overweight	Obesity	Overweight	Obesity
6	16.8	18.4	16.7	18.4
7	17.2	19.2	16.9	18.8
8	17.8	20.1	17.3	19.5
9	18.5	21.1	17.9	20.4
10	19.3	22.2	18.7	21.5
11	20.1	23.2	19.6	22.7

## Data Availability

No data were used to support this study.
